# Deep Transfer Learning Technique for Multimodal Disease Classification in Plant Images

**DOI:** 10.1155/2023/5644727

**Published:** 2023-05-13

**Authors:** V. Balaji, N. K. Anushkannan, Sujatha Canavoy Narahari, Punam Rattan, Devvret Verma, Deepak Kumar Awasthi, A. Anbarasa Pandian, M. R. M. Veeramanickam, Molla Bayih Mulat

**Affiliations:** ^1^Department of EEE, Aditya Engineering College, Surampalem, Andhra Pradesh, India; ^2^Department of ECE, Kathir College of Engineering, Coimbatore, Tamilnadu, India; ^3^Department of ECE, Sreenidhi Institute of Science and Technology, Hyderabad, Telangana, India; ^4^School of Computer Applications, Lovely Professional University, Phagwara, Punjab, India; ^5^Department of Biotechnology, Graphic Era Deemed to be University, Dehradun, 248002, Uttarakhand, India; ^6^IFTM University, Moradabad, Uttar Pradesh, India; ^7^Department of Computer Science and Engineering, Panimalar Engineering College, Poonamallae, Chennai, Tamilnadu, India; ^8^Centre of Excellence for Cyber Security Technologies, Institute of Engineering and Technology, Chitkara University, Chandigarh, Punjab, India; ^9^Department of Chemical Engineering College of Biological and Chemical Engineering, Addis Ababa Science and Technology University, Addis Ababa, Ethiopia

## Abstract

Rice (*Oryza sativa*) is India's major crop. India has the most land dedicated to rice agriculture, which includes both brown and white rice. Rice cultivation creates jobs and contributes significantly to the stability of the gross domestic product (GDP). Recognizing infection or disease using plant images is a hot study topic in agriculture and the modern computer era. This study paper provides an overview of numerous methodologies and analyses key characteristics of various classifiers and strategies used to detect rice illnesses. Papers from the last decade are thoroughly examined, covering studies on several rice plant diseases, and a survey based on essential aspects is presented. The survey aims to differentiate between approaches based on the classifier utilized. The survey provides information on the many strategies used to identify rice plant disease. Furthermore, model for detecting rice disease using enhanced convolutional neural network (CNN) is proposed. Deep neural networks have had a lot of success with picture categorization challenges. We show how deep neural networks may be utilized for plant disease recognition in the context of image classification in this research. Finally, this paper compares the existing approaches based on their accuracy.

## 1. Introduction

Plant disease detection is vital in agriculture because farmers must frequently assess whether the crop they are harvesting is suitable. It is critical to take these seriously because they can cause major difficulties in plants, affecting product quality, quantity, or productivity. Plant diseases generate disease outbreaks on a regular basis, resulting in large-scale death, and a negative impact on the economy. These issues must be addressed early on in order to save people's lives and money. Automatic classification of plant diseases is an essential study topic because it is critical in monitoring huge fields of crops and detecting disease indications on plant leaves at an early stage. Image-based automatic inspection can now be provided using computer vision algorithms. Manual identification, on the other hand, is labor demanding, less accurate, and can only be done in small regions at a time. This strategy allows plant diseases to be identified early on, and pest and infection management technologies can be utilized to solve pest problems while reducing dangers to people and the environment. When dealing with rice illnesses, there are several crucial factors to consider, including correct data gathering, proper rice plant monitoring, and many more. One of the most crucial and necessary stages is to collect samples from the sick rice plant. This can be accomplished by placing multimedia sensors across the property. This aids in the regular monitoring of the rice plant. Climate change and its impact on the rice plant can also be recorded and examined. However, this technology has some disadvantages, such as the need for regular system maintenance and the presence of a shadow in the photos acquired, which results in low accuracy. In the early detection of plant disease classifications in the form of a variety of species, many techniques and algorithms are used to detect and prevent entire diseases and classify the accuracy in the form enhanced way.

The early detection of the entire network is might more important one, thus many machine learning algorithms and fuzzy-based techniques are failures to describe the networks in the form of the early detection of the images.

Thus our paper focuses on the early detection of the network in the form of using various techniques and algorithms; this method of technology provides enhanced accuracy when compared with the many other existing techniques.

## 2. Objectives

The main objective of our paper provides that the early detection of plant diseases classifications in the form of multiple varieties of species, thus our paper proposed that deep learning methods help to detect the early detection of the entire networks. The preprocessing techniques help to detect the noise and the reduction of the noise and the feature extraction extract the whole image into pixel and convert these pixels into more manageable groups. The classification techniques using deep learning multiple convolutional neural networks provide enhanced accuracy when compared with the existing techniques.

## 3. Review of Literature

Shrivastava et al. [1] implemented the rice plant diseases classification using transfer learning of a deep convolutional neural network, this paper implements the rice plant disease classifications in the entire network, and the system this paper provides that the four types of the rice plant varieties in the entire networks, thus it provides that the rice blast, bacterial leaf blight, sheet blight, and the healthy leaf in the entire network system and then the classifications techniques involved in the form of the convolutional neural network and the feature extraction techniques take places in the form of the support vector machines.

Aderghal et al. [2] implemented the classifications of Alzheimer's diseases on imaging modalities with deep CNNs using cross-modal transfer learning. This paper proposes that the cross-model transfer learning, this method of accuracy detection provides enhanced ways, and finally, this paper compares with the existing approaches based on its accuracy and the classifications techniques may be handled in the form of the convolutional neural network.

Abdalla et al. [3] implemented the fine-tuning convolutional neural network with the transfer learning for semantic segmentation of ground-level oilseed rape images in a field with high weed pressure, the image segmentation is considered as the single step for the entire network and then the given datasets are worked with the visual geometry group (VGG)-19 methods; these datasets are pretrained by using the various methods in the form of the deep learning convolutional neural network. Finally, their paper provides the enhanced accuracy output when compared with the VGG-16 approaches.

Ghazi et al. [4] implemented that plant identification using deep neural convolutional neural network in the form of the transfer learning function that is why this paper provides the enhanced accuracy detection functions in the entire network and thus the network performance provides different classifiers and variety of datasets functions in the form of the enhanced accuracy output functions in the entire network. Finally, their paper compares with the existing approaches based on its accuracy.

Arshad et al. [5] implemented plant diseases identification using transfer learning; their paper implemented the multimodal convolutional neural network (MCNN) for the scratch and this approach is used for the enhancement of the accuracy. The datasets are pretrained by using the MCNN techniques than the feature extraction function, which helps to predict the better accuracy functions in the form of the classifications techniques. Finally, their paper provides that the enhanced accuracy when compared with the existing techniques.

Yuan et al. [6] implemented the advanced agricultural disease image recognition technologies in the form of a review. Their paper states that artificial intelligence provides a more challenging scheme in the entire network and that is why their paper provides the enhanced accuracy and the error detection function by using the deep learning and the transfer learning techniques. In the normal way, the artificial intelligence faces the most challenging one in the form of the many face detection. Finally, this paper compares with the existing approaches based on its accuracy.

Das et al. [7] implemented the automated classifications of cells into multiple classes in epithelial tissue of oral squamous cell carcinoma using transfer learning and a convolutional neural network. This paper proposed that in the deep learning convolutional neural network, many researchers were involved to detect the functions of the disease classifications in many approaches but they could not predict the early detection and the accuracy of evaluation in the entire network. And, finally, this paper provides enhanced accuracy detection when compared with the existing approaches.

Rajasekar et al. [8] implemented that the detection of cotton plant diseases using deep transfer learning; the agriculture is considered the most crucial part of the Indian growth and the economic development in each and every country thus it provides the food all over India. Thus the early detection and the prevention of the plant diseases is more crucial. One of our approaches provides that the enhanced accuracy detection and the noise removal in the uses of perfect deep learning convolutional neural network and then the preprocessing techniques. Their paper provides the enhanced accuracy outputs when compared with the existing approaches.

Garg et al. [9] implemented a multimodal system for precision agriculture using Internet of Things (IoT) and machine learning techniques; the way of increasing the crop production in the entire networks of agricultural farming is to reduce the entire plant disease by the use of the variety of techniques and the algorithm and, then it produces the enhanced quantity and quality of the things supplied in the form of the enhanced way. Finally, their paper implements the enhanced accuracy when compared with the existing techniques.

Sabatelli et al. [10] implemented the deep transfer learning for art classifications problems; this paper provides that the multimodal plant diseases classifications in the form of the various approaches and this paper implemented that the deep learning convolutional neural network and the feature extraction has been worked with the function of the soft-max classifier. Finally, this paper compares with the existing approaches based on its accuracy.

Too et al. [11] implemented the comparative study of fine-tuning deep learning models for plant diseases identifications. Recent days deep learning provides the fast and accurate detection of plant diseases classifications in the form of the recognition of various types of plants and its diseases. Our proposed methods provide that VGG-19 is used for the extraction of various amount of species and the layers in the entire network and the system. Finally it provides the enhanced accuracy detection when compares with the existing approaches.

Kora et al. [12] implemented the transfer learning techniques for medical images analysis in the review form. Their paper implements the transfer-learning methods for the identification of the data samples and the classification of the diseases using various methods and algorithm; the feature extraction helps in the early detection of the diseases. Finally, their paper provides enhanced accuracy outputs. At last, this paper compares the existing approaches based on their accuracy.

Zhao et al. [13] implemented the augmenting crop detection for precision with deep visual transfer learning, in the form of the case study of bale detection. Their paper implements the unmannered aerial vehicle (UAV) methods for the image identification and the classification methods, thus this methods helps to protect the enhanced accuracy outputs in the form of the various classifications and the feature extraction using the various attack detection methods. These methods provides that the enhanced accuracy detection when compared with the existing techniques.

Sowmya et al. [14] implemented the remote sensing satellite image processing techniques for image classifications. Their paper implements the leaf diseases classifications in the form of the four basic applications: image preprocessing, enhancement, transformation, and the classifications functions. This classification function helps to selected the pixels and provides better accuracy in the entire image processing system.

Lu and Weng [15] implemented the survey of image classifications methods and techniques for improving classifications performance. Their paper implements the image classifications based on the geographical information system, the nonparametric classifications techniques such that the neural network, decision tree classifier, and knowledge-based classification techniques; this technique provides that the enhanced accuracy. Finally, this paper compares the accuracy-based classifications in the existing techniques.

Huang et al. [16] implemented that the automatic labeling and selection of training samples for high-resolution remote sensing image classifications over urban areas, the leaf diseases classifications are more crucial to detect the accuracy results of the classifications of the plant diseases, thus their paper proposed the enhanced accuracy when compared with the existing approaches.

Hermosilla et al. [17] implemented the assessing contextual descriptive features for the plot-based classifications of urban areas. Their paper proposes that the geospatial datasets and the classifications techniques handled by using the plot-based image classifications and the feature extractions can be handled in the form of the various methods and then the outputs of the plant diseases classification in the form of the enhanced methods. Finally, their paper compares with the existing approaches.

Goldblatt et al. [18] implemented the detection of the boundaries of urban areas in India. Their paper provides that the google earth engine performs three types of classifiers, and the output of the total image processing provides enhanced accuracy outputs when compared with the other existing techniques.

Weng [19] implemented the remote sensing of impervious surfaces in the urban areas based on its requirements, methods, and trends. Their paper proposed that the artificial neural network (ANN) for the classifications of the given datasets and remote sensing methods used to extract the features in the entire image processing. Their paper provides the environment and the public sector datasets in the form of high-processing data.

Ehsanirad [20] implemented the plant diseases classifications based on leaf recognition; their paper implements that the two methods principle component analysis methods and the gray level cooccurrence matrix help to detect the classifications of the given datasets, and the classification approach provides 13 kinds of the plants and 65 species amounts in the entire image processing systems. Finally, this paper compares with the existing techniques.

Wang et al. [21] implemented the automatic image-based plant disease severity estimation using deep learning; the plant diseases classifications and the identifications are might more crucial one, thus their paper implements the deep learning convolutional neural network for the accuracy and the classification detection. Their paper implements the VGG-16 model for the techniques of the classification of the accuracy detection in the entire images processing leaf class classifications.

DeChant et al. [22] implemented the automated identifications of northern leaf blight-infected maize plants from field imagery using deep learning. This paper implements that the northern leaf blight causes severe problem in the entire maize plants, thus their paper implements the deep learning convolutional neural network, and the dataset are trained by the heat map giving enhanced throughput power and without the use of the pesticides providing the enhanced accuracy output in this types of the concept.

Singh et al. [23] implemented the deep learning for plant stress phenotyping: trends and future perspectives. Their paper compares the machine learning and the deep learning techniques based on the large amounts of the given datasets, and the procedure may depend upon the phenotype and the genotype methods, thus it provides enhanced throughput and accuracy power in the entire networking system.

Gonçalves et al. [24] implemented the deep learning architectures for semantic segmentation and automatic estimation of the severity of foliar symptoms caused by diseases or pests. Their paper states that the color thresholding digital image processing methods help to identify the severe quality of the plant diseases and that deep learning convolutional neural network helps to classify the images based on the classification of the disease. Their paper implemented six layers of the convolutional layer that help to detect and rectify the fungal disease classification in the plants and further enhanced accuracy in the entire image processing.

Nagasubramanian et al. [25] implemented the plant disease identifications using explainable 3D deep learning on hyperspectral images. Their paper implemented the hyperspectral image processing in the entire deep convolutional neural network, thus their paper provides enhanced accuracy and throughput power in the entire network system.

## 4. Overview of Proposed Methods

The overview of the proposed methods provides the basic functions of the image processing techniques. For the classification, we applied the concept of transfer learning. The key advantage of employing transfer learning is that instead of starting from scratch, the model starts from patterns learned when tackling a different problem that is similar in nature to the one being solved. In this manner, the model builds on existing knowledge rather than starting from scratch. Transfer learning is typically expressed in image classification through the use of pretrained models. A pretrained model is one that has been trained on a big benchmark dataset to tackle a problem comparable to the one we wish to solve. For our work, we employed two pretrained models, ResNet-50 and VGG-16, as pretrained weights. The enhanced multiple convolutional neural network with genetic algorithm consists of five convolutional layers, and each section is followed by the Relu layer, which helps to minimize the error in the entire network and the batch normalization in the form of the normalizing in the form of the functions, and the three max pooling layer provides that the fully connected layer with the form of the softmax activation. The feature extraction techniques use a genetic algorithm, while the classification procedures are handled by many types of deep learning convolutional neural networks, resulting in improved detection accuracy when compared with previous methodologies.

Figure 1 implements the overview of the proposed methods, the proposed methods provide that the entire image processing techniques, like this technique, contain the preprocessing, which helps to reduce the noise in the entire image, and the feature extraction is handled by using the genetic algorithm; the classification techniques are involved in the form of the enhanced convolutional neural network.

### 4.1. Proposed Approach

Figure 2 implements the proposed approaches, and the proposed methods contain the further approaches used in the proposed paper. Our paper provides the preprocessing techniques based on the Gaussian filter; this filter helps to reduce the noise in the filter and converts the images into RGB to greyscale images. After the completion of the preprocessing techniques, the feature extraction techniques take place. Our paper proposes that the genetic algorithm for the feature extraction provides enhanced accuracy detection, and it helps to classify the better accuracy detection in the entire networks. Finally the classification techniques take places, and our paper proposed the enhanced convolutional neural network for the classifications approaches.

### 4.2. Preprocessing

The preprocessing technique is considered one of the most crucial techniques, thus it helps to detect the noise in the network by adding some of the filters that help to reduce the noise in the entire image processing network. Our paper implements that the Gaussian filter helps to reduce the noise in the entire image processing network. Finally, this paper provides the error-free function in the entire network. The normal functions of the preprocessing reduced the noise in the entire image processing and the conversion of the images into (red green blue) RGB to the gray level images. Then the final results of the images are converted into better-enhanced outputs [26–32].

The Gaussian filter is considered the linear filter; it helps to reduce the blur in the images, and then the results of the Gaussian images may be used as the unsharp masking since it can be used as the edge detection function.

Thus the Gaussian filter is considered as the low pass filter, and the mathematical expression for this filter is considered as

(1) $$\begin{array}{c} G\left(u,s\right)=\frac{1}{2\times 3.14\partial^{2}}e^{\left(-u^{2}+s^{2}\right)/2\partial^{2}}. \end{array}$$

The *u* and *s* are considered as the coordinate value and then the *∂* is denoted as the standard deviation respectively.

### 4.3. Genetic Algorithm

The genetic algorithm provides that gene functions help to detect the plant diseases detection in the form of the urban plant diseases classifications. It contains mainly three functions.

Figure 3 represents the genetic algorithm in the form of the apple plant disease classifications. The genetic algorithm is one of the most crucial ones to detect the extraction of the features in the image processing, the better accuracy results in the image processing only depends on the feature extractions.

Every pixel inside the images depends on the adjacent pixel range, and it provides a better quality of the images.

The very first process of the genetic algorithm is to predict and select the best points in the image functions and then it performs the overfitting functions. Thus the final part of the session provides the adding sequence in the entire image processing. The genetic algorithm only depends on the fitness function in the entire system.

The genetic algorithm is based on three functions namely operation in the selection, operation in cross over, and the operation in the mutation function.

These genetic functions based on the overfitting functions. It helps to reduce the overfitting functions in the image processing. This output result gives the input for the classification techniques.

### 4.4. Transfer Learning

As we all know that the deep learning model provides enhanced accuracy outputs when compared with the existing techniques and it helps to solve many complex problems in the entire plant disease classifications. It helps to build the pretrained image segmentation functions. The ResNet-50 with pretrained functions is used to extract the features by using the form of the fully connected layer and then this analysis provides the enhanced form of the result in the form of the Softmax functions. And, finally, the comparison methods may be established in the form of the VGG-16 functions, and then the fully connected layer and the softmax layers provide more number of possible neurons.

### 4.5. Enhanced Multiple Convolutional Neural Network

The enhanced multiple convolutional neural network architecture consists of five convolutional layers and thus each section is followed by the Relu layer; the Relu layer helps to minimize the error in the entire network and the batch normalization in the form of the normalizing in the form of the functions. The three max pooling layer provides the fully connected layer with the form of the Softmax activation [1].

(2) $$\begin{array}{c} \text{Sensitivity}=\frac{TP}{TP+FN}\times 100, \end{array}$$

(3) $$\begin{array}{c} \text{Specificity}=\frac{TN}{TN+FP}\times 100, \end{array}$$

(4) $$\begin{array}{c} \text{Accuracy}=\frac{TN+TP}{TN+TP+FN+FP}\times 100, \end{array}$$

(5) $$\begin{array}{c} \text{Index}=\text{Sensitivity}+\text{Specificity}-1. \end{array}$$

The above equations show the sensitivity, specificity, accuracy, and index obtained from the given datasets.

## 5. Datasets

Our paper implements the benchmark public collections of the datasets and then these techniques provide that ResNet-50 and the VGG-16 help to extract the features with the help of many functions. The datasets are preprocessed by the Gaussian filter, and the rice crop provides that enhanced accuracy detection methods form because the Gaussian filter helps to reduce the whole noise and attacks in the images and also reduces the blurring effects in the entire network by the use of the data augmentation in the entire image processing. The genetic algorithm helps to reduce the noise in the entire image processing and provides the enhanced extraction of the features in the entire image processing. Our paper implements that the enhanced multiple convolutional neural networks for detecting better accuracy using these methods.

## 6. Comparison Analysis and Results

Our paper proposed the formation of the plant diseases classifications in the form of the multimodal variety; thus our paper provides that the data augmentation and the Gaussian filter for the preprocessing techniques and the genetic algorithm functions for the feature extraction and the classification techniques handled by using the enhanced convolutional neural networks.

Figure 4 provides the enhanced accuracy of plant disease classifications in the form of comparison results.

## 7. Conclusion and Future Work

Rice disease is the most common problem for most farmers, so early detection is critical. With advances in science, identifying rice illness is considerably easier than it was in the past, when manual inspection was used. Based on the classifier utilized, this study report summarized numerous strategies for identifying rice illnesses. It was also discovered that the CNN classifier excels at pattern recognition, which is a fundamental notion in image processing. Our suggested model, which is based on CNN, offers promising results in terms of accuracy. The purpose of this research is to illustrate the technological viability of deep learning utilizing a convolutional neural network approach to enable autonomous disease detection via image classification. Our paper proposed the rice plant diseases classifications in the form of multimodal methods, in which the collective datasets are gathered to the preprocessed function, and our preprocessing methods are handled in the form of the Gaussian filter. The feature extraction techniques work with the genetic algorithm, and then the classification techniques are handled by the multiple forms of deep learning convolutional neural network, providing enhanced accuracy. Our future studies will address the form of the genetic algorithm using upgraded support vector machine techniques.

## Figures and Tables

**Figure 1:** Overview of the proposed approach.

**Figure 2:** Proposed approach.

**Figure 3:** Genetic algorithm.

**Figure 4:** Results.

## Data Availability

The datasets used and/or analyzed during the current study are available from the corresponding author upon reasonable request.

## References

[1] Shrivastava V. K., Pradhan M. K., Minz S., Thakur M. P. (2019). Rice plant disease classification using transfer learning of deep convolution neural network. *The International Archives of the Photogrammetry, Remote Sensing and Spatial Information Sciences*.

[2] Aderghal K., Khvostikov A., Krylov A., Benois-Pineau J., Afdel K., Catheline G. Classification of Alzheimer disease on imaging modalities with deep CNNs using cross-modal transfer learning.

[3] Abdalla A., Cen H., Wan L. (2019). Fine-tuning convolutional neural network with transfer learning for semantic segmentation of ground-level oilseed rape images in a field with high weed pressure. *Computers and Electronics in Agriculture*.

[4] Ghazi M. M., Yanikoglu B., Aptoula E. (2017). Plant identification using deep neural networks via optimization of transfer learning parameters. *Neurocomputing*.

[5] Arshad M. S., Rehman U. A., Fraz M. M. Plant disease identification using transfer learning.

[6] Yuan Y., Chen L., Wu H., Li L. (2022). Advanced agricultural disease image recognition technologies: a review. *Information Processing in Agriculture*.

[7] Das N., Hussain E., Mahanta L. B. (2020). Automated classification of cells into multiple classes in epithelial tissue of oral squamous cell carcinoma using transfer learning and convolutional neural network. *Neural Networks*.

[8] Rajasekar V., Venu K., Jena S. R., Varthini R. J., Ishwarya S. (2021). Detection of cotton plant diseases using deep transfer learning. *Journal of Mobile Multimedia*.

[9] Garg S., Pundir P., Jindal H., Saini H., Garg S. Towards a multimodal system for precision agriculture using IoT and machine learning.

[10] Sabatelli M., Kestemont M., Daelemans W., Geurts P. Deep transfer learning for art classification problems.

[11] Too E. C., Yujian L., Njuki S., Yingchun L. (2019). A comparative study of fine-tuning deep learning models for plant disease identification. *Computers and Electronics in Agriculture*.

[12] Kora P., Ooi C. P., Faust O. (2022). Transfer learning techniques for medical image analysis: a review. *Biocybernetics and Biomedical Engineering*.

[13] Zhao W., Yamada W., Li T., Digman M., Runge T. (2021). Augmenting crop detection for precision agriculture with deep visual transfer learning—a case study of bale detection. *Remote Sensing*.

[14] Sowmya D. R., Shenoy P. D., Venugopal K. R. (2017). Remote sensing satellite image processing techniques for image classification: a comprehensive survey. *International Journal of Computer Applications*.

[15] Lu D., Weng Q. (2007). A survey of image classification methods and techniques for improving classification performance. *International Journal of Remote Sensing*.

[16] Huang X., Weng C., Lu Q., Feng T., Zhang L. (2015). Automatic labelling and selection of training samples for high-resolution remote sensing image classification over urban areas. *Remote Sensing*.

[17] Hermosilla T., Ruiz L. A., Recio J. A., Cambra-López M. (2012). Assessing contextual descriptive features for plot-based classification of urban areas. *Landscape and Urban Planning*.

[18] Goldblatt R., You W., Hanson G., Khandelwal A. K. (2016). Detecting the boundaries of urban areas in india: a dataset for pixel-based image classification in google earth engine. *Remote Sensing*.

[19] Weng Q. (2012). Remote sensing of impervious surfaces in the urban areas: requirements, methods, and trends. *Remote Sensing of Environment*.

[20] Ehsanirad A. (2010). Plant classification based on leaf recognition. *International Journal of Computer Science and Information Security*.

[21] Wang G., Sun Y., Wang J. (2017). Automatic image-based plant disease severity estimation using deep learning. *Computational Intelligence and Neuroscience*.

[22] DeChant C., Wiesner-Hanks T., Chen S. (2017). Automated identification of northern leaf blight-infected maize plants from field imagery using deep learning. *Phytopathology*.

[23] Singh A. K., Ganapathysubramanian B., Sarkar S., Singh A. (2018). Deep learning for plant stress phenotyping: trends and future perspectives. *Trends in Plant Science*.

[24] Gonçalves J. P., Pinto F. A. C., Queiroz D. M., Villar F. M. M., Barbedo J. G. A., Ponte E. M. D. (2021). Deep learning architectures for semantic segmentation and automatic estimation of severity of foliar symptoms caused by diseases or pests. *Biosystems Engineering*.

[25] Nagasubramanian K., Jones S., Singh A. K., Sarkar S., Singh A., Ganapathysubramanian B. (2019). Plant disease identification using explainable 3D deep learning on hyperspectral images. *Plant Methods*.

[26] Rathish C. R., Rajaram A. (2016). Efficient path reassessment based on node probability in wireless sensor network. *International Journal of Control Theory and Applications*.

[27] Basha S. R., Sharma C., Sayeed F. (2022). Implementation of reliability antecedent forwarding technique using straddling path recovery in manet. *Wireless Communications & Mobile Computing*.

[28] Rathish C. R., Rajaram A. (2015). Hierarchical load balanced routing protocol for wireless sensor networks. *International Journal of Applied Engineering Research*.

[29] Rajaram A., Sathiyara K. (2022). An improved optimization technique for energy harvesting system with grid connected power for green house management. *Journal of Electrical Engineering & Technology*.

[30] Dinesh M., Arvind C., Mole S. S. S. (2022). An energy efficient architecture for furnace monitor and control in foundry based on industry 4.0 using IoT. *Scientific Programming*.

[31] Mahalakshmi K., Kousalya K., Shekhar H. (2021). Public auditing scheme for integrity verification in distributed cloud storage system. *Scientific Programming*.

[32] Divakaran J., Malipatil S., Zaid T. (2022). Technical study on 5G using soft computing methods. *Scientific Programming*.

